The article "Clinical Impact of Nurses-Physicians Collaboration Intervention on the Treatment of Immune Recurrent Spontaneous Abortion with Low-Molecular-Weight Heparin" was retracted in 2023. Reasons: unreliable results or conclusions; concerns about the data; concerns about the peer review; concerns about the citations.

# Clinical Impact of Nurses-Physicians Collaboration Intervention on the Treatment of Immune Recurrent Spontaneous Abortion with Low-Molecular-Weight Heparin

**DOI:** 10.1155/2021/9290720

**Published:** 2021-10-29

**Authors:** Miaocheng Chen, Xi Wang, Peiru Deng

**Affiliations:** Department of Obstetrics, Huizhou Central People's Hospital, Huizhou, Guangdong 516000, China

## Abstract

Anticoagulation is currently the preferred and effective treatment for patients with recurrent spontaneous abortion (RSA), but, due to the prevalence of mood disorders in RSA patients and the high number of adverse effects associated with long-term medication, effective care measures are often required. In this study, 94 patients with immune-type RSA who were admitted to our hospital from January 2018 to June 2019 were selected and randomly divided into a control group and a study group of 47 patients each; both groups received low-molecular-weight heparin treatment after admission, and the control group received conventional nursing interventions during treatment, while the patients in the study group received integrated medical and nursing care interventions. Pregnancy outcomes, pre- and postintervention scores on the Self-Assessment Scale (SAS), Self-Depression Scale (SDS), and Pittsburgh Sleep Quality Index (PSQI), levels of serum gamma-interferon (IFN-*γ*) and interleukin-4 (IL-4) and their ratios, complications, and patient satisfaction with the intervention were observed in both groups. The results showed that the success rate of fetal preservation in the study group (89.36%) was significantly higher than that in the control group (68.09%) (*P* < 0.05). After treatment, SAS, SDS, and PSQI scores decreased in both groups, with the study group being lower (*P* < 0.05). IFN-*γ* and IFN-*γ*/IL-4 levels decreased and IL-4 levels increased in both groups after treatment, with IFN-*γ* and IFN-*γ*/IL-4 being significantly lower and IL-4 levels being significantly higher in the study group than in the control group (*P* < 0.05). The incidence of adverse drug reactions in the study group was significantly lower than that in the control group (*P* < 0.05). Patients in the study group were more satisfied with all aspects of the intervention than the control group (*P* < 0.05). These results suggest that nurses-physicians collaboration intervention may improve the effectiveness of low-molecular-weight heparin therapy in patients with immune-type RSA. It helps to improve patient pregnancy outcomes, mood, sleep quality, and immune function and increases patient satisfaction.

## 1. Introduction

Recurrent spontaneous abortion (RSA) is a condition in which a woman of childbearing age suffers two or more consecutive spontaneous abortions with the same sexual partner, with prevalence of approximately 1% to 5% of women of childbearing age [1]. The etiology of RSA is complex and relatively clear causes include chromosomal abnormalities, endocrine system factors, reproductive tract infections, immune factors, and prethrombotic states, among which RSA due to immune imbalance, that is, immune-type RAS, is one of the main types of the disease [2]. The mechanism of action of clinically used low-molecular-weight heparin on RAS is unclear and may be related to its immunosuppressive and immunomodulatory properties. It may promote embryonic growth and development by improving maternal blood hypercoagulability, reducing blood viscosity and vascular resistance, increasing placental blood supply, and fundamentally altering intrauterine microcirculation [3, 4].

The article "Clinical Impact of Nurses-Physicians Collaboration Intervention on the Treatment of Immune Recurrent Spontaneous Abortion with Low-Molecular-Weight Heparin" was retracted in 2023. Reasons: unreliable results or conclusions; concerns about the data; concerns about the peer review; concerns about the citations.

A study on the psychological state of RSA patients found that the prevalence of negative emotions such as anxiety and depression was generally high among RSA patients [5]. The greater the number of miscarriages, the greater the risk of miscarriage in further pregnancies, leading to a gradual increase in the psychological pressure of fear of pregnancy failure and a tendency to lose confidence in pregnancy, with patients often displaying psychological states such as depression and sadness [6]. The stimulation of negative emotions such as excessive anxiety and depression can put the body in a hyperactive state and affect the normal development of the embryo through the overreaction of various regulatory mechanisms, which can lead to adverse pregnancy outcomes such as intrauterine growth restriction, intrauterine death, miscarriage, and preterm delivery [7, 8]. Moreover, some patients may not cooperate with treatment and interrupt treatment during the treatment process due to the influence of emotions, thus affecting the treatment effect. Clinical studies have shown that low-molecular-weight heparin is effective in the treatment of immune RSA, but the treatment of immune RSA is not limited to the rational use of drugs as it also requires effective nursing measures [9]. The nurses-physicians collaboration intervention model refers to a relatively fixed treatment team of doctors and nurses to provide patients with integrated treatment, nursing care, and rehabilitation services, which can achieve the effect of “1 + 1>2” [10]. The studies in [11, 12] have shown that the nurses-physicians collaboration intervention model can improve the quality of medical safety, enhance the awareness of medical and nursing cooperation, and improve the level of medical and nursing cooperation, but there is a lack of research on the integrated medical and nursing cooperation model in the care of immune-type RSA during treatment.

The article "Clinical Impact of Nurses-Physicians Collaboration Intervention on the Treatment of Immune Recurrent Spontaneous Abortion with Low-Molecular-Weight Heparin" was retracted in 2023. Reasons: unreliable results or conclusions; concerns about the data; concerns about the peer review; concerns about the citations.

In this study, we give full play to the advantages of integrated nurses-physicians collaboration during the treatment of immune RSA patients via low-molecular-weight heparin, standardize the nursing process, and strengthen the communication and medical and nursing cooperation. The study's application was evaluated using indicators of fetal preservation success, emotional status, sleep status, immune function, and patient satisfaction to explore its feasibility and applicability and to provide a practical basis for nursing research during treatment of immune-type RSA.

## 2. Materials and Methods

### 2.1. Materials

94 patients with immune RSA who were admitted to our hospital from January 2018 to June 2019 were selected for the study, with the patients' ages ranging from 22 to 40 years, with a mean of 30.41 ± 3.13 years. Patients were coded according to their order of admission in order of 1 to 94, and the enrolled patients were randomly divided into a control group and a study group of 47 cases each according to the random number table method. Patients in the control group were treated with conventional care and low-molecular-weight heparin, while those in the study group received nurses-physicians collaboration and low-molecular-weight heparin. General data such as age distribution, history of miscarriage, number of years of marriage, and week of gestation were collected and compared between the two groups and the differences were not statistically significant (*P* > 0.05, Table 1) and were comparable.

### 2.2. Diagnostic Criteria for RSA [13]

The diagnostic criteria for RSA were as follows: (1) patients having a history of menopause with no or a small amount of vaginal bleeding or with symptoms such as cramping in the abdomen and lumbar pain; (2) positive urine pregnancy test; (3) unopened cervical opening, soft uterine body, and uterine body size generally consistent with the number of days of menopause; (4) ultrasound examination confirming intrauterine pregnancy; and (5) ≥ 2 consecutive spontaneous abortions with the same sexual partner.

### 2.3. Inclusion Criteria

The inclusion criteria were as follows: (1) patients with RSA who received fetal preservation treatment after admission; (2) gestational age ≤12 weeks; (3) autoimmune antibody test: anti-cardiolipin antibody (ACA), anti-endometrial antibody (EMAb) in IgG, and IgM, at least one of which is weakly positive; (4) no previous history of stillbirth or live birth; and (5) patients being informed about the study and signing an informed consent form.

### 2.4. Exclusion Criteria

The exclusion criteria were as follows: (1) patients with recent spontaneous abortion, embryonic arrest, biochemical pregnancy, and other abnormal pregnancies; (2) patients who have taken drugs affecting immune function prior to admission or who have recently received immunotherapy; (3) patients with other immune diseases; (4) patients with more serious diseases of the heart, brain, liver, kidney, and haematopoietic system and psychiatric abnormalities; (5) patients with reproductive tract infections and malformations; (6) patients with abnormal coagulation function; (7) combination of other pregnancy complications such as severe pregnancy vomiting; and (8) failure to use the medication as prescribed and being unable to determine the efficacy or incomplete information affecting the efficacy.

The article "Clinical Impact of Nurses-Physicians Collaboration Intervention on the Treatment of Immune Recurrent Spontaneous Abortion with Low-Molecular-Weight Heparin" was retracted in 2023. Reasons: unreliable results or conclusions; concerns about the data; concerns about the peer review; concerns about the citations.

### 2.5. Treatment and Care Intervention Methods

Patients in both groups received low-molecular-weight heparin treatment upon admission: patients were given an abdominal subcutaneous injection of low-molecular-weight heparin calcium at a starting dose of 10,000 IU every 12 hours. The prothrombin time test was performed every 2 days during the treatment period, and the dose of medication was adjusted according to the test results. After the prothrombin time reaches about 1.5 times that of normal pregnant women, the ACA test was performed once a month, and the medication was stopped if the result was negative; the medication was resumed when the test result turned positive. The dose was reduced to 5000 IU per day after 6 months of initial treatment. The duration of treatment was based on fetal maturity and was usually discontinued at 34–36 weeks of gestation. Meanwhile, patients in the control group received routine care, including admission instructions, preparation for treatment, regular ward rounds, and medication care. The study group received integrated nurses-physicians collaboration intervention as follows:

1. Nurses-physicians collaboration care team was formed: it included the chief or deputy chief physician, the attending physician, the nurse, and the patient's family. Obstetricians and psychologists were also invited to provide professional training to the medical and nursing staff. The main contents of the training include the cooperation mode of medical and nursing staff in different stages of the disease, the way of communication with pregnant women, and psychological care.
2. Intervention programme was developed: patients were received by physicians and nursing staff together upon admission to the hospital, where they were asked about their medical history, and a treatment and care plan was developed. The patient's knowledge of RSA, the effects and prognosis of low-molecular-weight heparin treatment, nurses-physicians collaboration, and adverse drug reactions will greatly reduce the fear and anxiety of the unknown once the patient becomes familiar with the entire treatment process. The patient's psychological state and sleep status were assessed and the patient's need for and acceptance of integrated nursing care interventions were analysed to develop a personalised care plan.
3. Implementation of interventions: throughout the treatment process, the nurses-physicians collaboration care team needed to adjust synchronous shifts and synchronised room visits in order to be able to understand the patient's situation at the same time, and they also needed to communicate with the patient on a regular basis so that the patient understands her condition, the effect of treatment the specific measures taken, and so forth. The nurses-physicians team could adjust the treatment and care plan according to the specific situation and improve the patient's confidence so that she could face the treatment positively. For some patients with serious negative emotions, nursing staff should focus on psychological counselling and find effective breakthroughs in their family and social relationships. The injection site should be carefully examined before the injection treatment was carried out, the means of exhausting the injection should be improved, sterile cotton balls should be taken and pressed for about 3 minutes after the injection, and any bleeding tendencies or adverse drug reactions should be carefully asked and checked.

The article "Clinical Impact of Nurses-Physicians Collaboration Intervention on the Treatment of Immune Recurrent Spontaneous Abortion with Low-Molecular-Weight Heparin" was retracted in 2023. Reasons: unreliable results or conclusions; concerns about the data; concerns about the peer review; concerns about the citations.

### 2.6. Indicators of Observation

1. Effect on the success rate of fetal preservation and adverse reactions: observe and record the pregnancy outcomes such as full-term delivery, miscarriage, survival of preterm delivery, and death of preterm delivery in both groups, and calculate the success rate of fetal preservation as an indicator of efficacy. The success rate of fetal preservation = (survival of preterm birth + full-term birth) number of cases/total number of cases × 100%. The incidences of adverse reactions such as skin ecchymosis, haematoma, gastrointestinal discomfort, and thrombocytopenia were observed and recorded in both groups, and the overall incidence of adverse reactions was compared between the two groups.
2. Effects on patients' psychological status and sleep quality: before and after the intervention, patients' psychological status was assessed by Self-Rating Anxiety Scale (SAS) and Self-Rating Depression Scale (SDS), and sleep quality was assessed by Pittsburgh Sleep Quality Index (PSQI). The SAS and SDS consisted of 20 items, and the scores were rated according to the frequency of symptoms and were divided into 4 levels in order of 1, 2, 3, and 4. All scores were summed and multiplied by 1.25, rounded to the nearest whole number to obtain the standard score, and the higher the score, the greater the anxiety level. The SAS standard score cut-off was 50, where <50 was no anxiety, 50–59 was mild anxiety, 60–69 was moderate anxiety, and ≥70 was severe anxiety. The SDS standard score cut-off was 53, where <53 was no depression, 53–62 was mild depression, 63–72 was moderate depression, and ≥73 was severe depression [14]. The PSQI scale includes 23 entries in 7 components: sleep quality, time to fall asleep, sleep duration, sleep efficiency, sleep disorders, hypnotic drugs, and daytime function. Each component had a score of 0, 1, 2, or 3, and the cumulative component scores were total PASI scores, which ranged from 0 to 21, with higher scores suggesting poorer sleep quality in patients.
3. Effect on patients' immune function: 5 mL of fasting elbow venous blood was drawn on admission and after intervention in both groups, placed in anticoagulation tubes, and centrifuged at 3000 r·min^−1^ for 10 min, and the serum was collected and stored in a refrigerator at −70°C. The levels of serum gamma-interferon (IFN-*γ*) and interleukin-4 (IL-4) were measured by ELISA and the ratio of the two was calculated. The serum IFN-*γ* ELISA kit and serum IL-4 ELISA kit were purchased from Quanzhou Jiubang Biotechnology Co., and the relevant operation steps were carried out in strict accordance with the kit instructions.
4. Survey on patient satisfaction: the questionnaire was designed based on the relevant literature [15, 16] and included five dimensions of patients' satisfaction with the inpatient guidance, doctors, nursing staff, nurses and physicians cooperation, and doctor-patient communication, with four items in each dimension and an internal consistency Cronbach's alpha coefficient of 0.820. According to the degree of satisfaction, a 5-level scoring method is used: “very dissatisfied,” “unsatisfied,” “average,” “satisfied,” and “very satisfied” with 1 to 5 points. Each dimension has a score range of 4 to 20 and the total score range is 20 to 100, with higher scores indicating higher patient satisfaction.

The article "Clinical Impact of Nurses-Physicians Collaboration Intervention on the Treatment of Immune Recurrent Spontaneous Abortion with Low-Molecular-Weight Heparin" was retracted in 2023. Reasons: unreliable results or conclusions; concerns about the data; concerns about the peer review; concerns about the citations.

### 2.7. Statistical Methods

All data were processed using SPSS 22.0 statistical software and statistical graphs were produced using GraphPad Prism 8. The measurement data were expressed as mean ± standard deviation (mean ± SD) and independent-sample *t*-test was used for comparison between groups, and the count data were expressed as *n*, %, and *χ*^2^ test was used. Differences were indicated as statistically significant when *P* < 0.05.

## 3. Results

### 3.1. Comparison of Pregnancy Outcomes between the Two Groups

By recording and comparing the pregnancy outcomes of the two groups, we found that the proportions of full-term delivery, miscarriage, survival of preterm delivery, and death of preterm delivery in the control group were 38.30% (18 cases), 27.66% (13 cases), 19.15% (7 cases), and 19.15% (9 cases), respectively, with a success rate of 53.19% (25/47) of fetal preservation. The percentages of full-term delivery, miscarriage, survival of preterm delivery, and death of preterm delivery in the study group were 76.60% (36 cases), 8.51% (4 cases), 12.77% (6 cases), and 2.13% (91 cases), respectively, with a fetal preservation success rate of 89.36% (25/47). The success rate of pregnancy preservation was higher in the study group (89.36%) than in the control group (68.095), with a statistically significant difference (*P* < 0.05, Figure 1).

### 3.2. Comparison of Negative Mood Scores and Sleep Quality Scores before and after Intervention between the Two Groups

Negative emotion scores such as SAS and SDS as well as PSQI scores were assessed before and after the intervention in both groups and the data were compared. The results showed that there was no statistical difference between the SAS scores, SDS scores, and PSQI scores of the two groups before the intervention (*P* > 0.05). The SAS scores, SDS scores, and PSQI scores of both groups decreased after the intervention compared to the preintervention period, with the study group being lower than the control group and the difference being statistically significant (*P* < 0.05) (Figure 2).

### 3.3. Comparison of Immune Function Indexes before and after Intervention between the Two Groups

IFN-*γ* and IL-4 levels were measured before and after the intervention in both groups, and the IFN-*γ*/IL-4 ratio was calculated and the results were compared. The results showed that there was no statistical difference in the levels of IFN-*γ*, IL-4, and IFN-*γ*/IL-4 ratio between the two groups before and after the intervention (*P* > 0.05). The IFN-*γ* level and IFN-*γ*/IL-4 ratio decreased and the IL-4 level increased in both groups after the intervention; the IFN-*γ* level and IFN-*γ*/IL-4 ratio in the study group were lower than those in the control group, and the IL-4 level was higher than that in the control group, with the difference being statistically significant (*P* < 0.05) (Figure 3).

### 3.4. Comparison of Patient Satisfaction Survey Scores between the Two Groups

The patients' satisfaction with the effectiveness of medical care in the two groups was investigated and counted. The results showed that the study group was more satisfied than the control group in terms of satisfaction with the inpatient guidance, satisfaction with the doctors, satisfaction with the nursing staff, satisfaction with the cooperation between doctors and nurses, and satisfaction with the communication between doctors and patients, and the total score was also higher than that of the control group, with a statistically significant difference (*P* < 0.05) (Figure 4).

The article "Clinical Impact of Nurses-Physicians Collaboration Intervention on the Treatment of Immune Recurrent Spontaneous Abortion with Low-Molecular-Weight Heparin" was retracted in 2023. Reasons: unreliable results or conclusions; concerns about the data; concerns about the peer review; concerns about the citations.

### 3.5. Comparison of the Incidence of Adverse Drug Reactions between the Two Groups

By counting and analysing the occurrence of adverse reactions in the two groups during treatment, the results showed that the incidences of adverse reactions such as skin ecchymosis, haematoma, gastrointestinal discomfort, and thrombocytopenia in the control group were 8.51% (4 cases), 4.26% (2 cases), 8.51% (4 cases), and 10.64% (5 cases), respectively, and the overall incidence of adverse reactions was 31.91% (15/47). The incidences of adverse reactions such as skin petechiae, haematoma, gastrointestinal discomfort, and thrombocytopenia in the study group were 2.13% (1 case), 2.13% (1 case), 4.26% (2 cases), and 4.26% (2 cases), respectively, with an overall adverse reaction rate of 12.77% (6/47). The incidence of total adverse reactions in the study group was lower than that in the control group, and the difference was statistically significant (*P* < 0.05, Figure 5).

## 4. Discussion

RSA has high prevalence in women of childbearing age and is a clinically complex and difficult-to-treat condition that has become a hot issue in modern medical research. It can be caused by a variety of factors such as maternal endocrine disorders, reproductive tract abnormalities, and immune function, of which immune function abnormalities are the more common cause of RSA [17]. RSA due to abnormal immune function, also known as immune-type RSA, is clinically treated with low-molecular-weight heparin, which is effective in improving the symptoms of abnormal immune function in patients [18]. However, due to multiple miscarriages, RSA patients tend to suffer from anxiety and depression, and the long-term application of low-molecular-weight heparin can lead to adverse effects such as skin ecchymosis, causing or aggravating psychological trauma in patients [19]. As a result, treatment alone is not comprehensive enough for RSA patients and needs to be accompanied by appropriate nursing interventions. The current disease-centred conventional care no longer meets the needs of patients and an integrated patient-centred nursing intervention model has emerged.

Treatment and nursing are two closely related but relatively independent systems in medical work. Traditionally, medical and nursing work is carried out independently, with nurses carrying out medical orders after doctors have given them, and nurses do not participate in doctors' morning check-ups, leading to insufficient communication between nurses and doctors and easily causing negligence in all aspects, which has a negative impact on follow-up work and the patient's disease regression [20, 21]. The implementation of the integrated management model of nurses-physicians collaboration breaks the pattern of two parallel lines of doctor-patient and nurse-patient under the traditional model of nursing care and rebuilds a new working pattern of the trinity of doctor, nurse, and patient to achieve the maximum effect of nursing interventions [22]. In a survey of nine intensive care units, Wang et al. [23] showed that nurse-physician collaboration helped to reduce the incidence of postoperative infections in critically ill patients, shorten treatment time, and facilitate the recovery process and that active nurse-physician collaboration improved nurse job satisfaction, increased identification with the team, and reduced turnover intentions. Williams et al. [24] showed that a collaborative physician-nurse intervention model for geriatric patients in outpatient clinics could provide high-quality care and improve patient satisfaction without increasing healthcare costs. In this study, on the basis of low-molecular-weight heparin treatment for immune-type RSA patients, integrated physicians and nursing care interventions such as simultaneous reception of patients, assessment of patients' conditions, development of care plans, health education, and ward rounds were used. The results showed that the success rate of fetal preservation was higher in the study group than in the control group, and the incidences of SAS, SDS, PSQI scores, and adverse reactions were significantly lower in the study group than in the control group after the intervention. It was suggested that the improvement of psychological negative emotions and sleep quality in the integrated medical care patient group was better than that in the conventional care group, and the incidence of adverse drug reactions was reduced. To analyse the reasons, detailed health education and psychological communication by medical and nursing staff in the integrated care model can improve the psychological status of patients, thus increasing treatment compliance and improving treatment outcomes. In addition, the detailed health education improved the patients' ability of self-testing and management and avoided the occurrence of abnormal reactions, so the incidence of adverse reactions in the study group was significantly lower than that in the control group.

The article "Clinical Impact of Nurses-Physicians Collaboration Intervention on the Treatment of Immune Recurrent Spontaneous Abortion with Low-Molecular-Weight Heparin" was retracted in 2023. Reasons: unreliable results or conclusions; concerns about the data; concerns about the peer review; concerns about the citations.

The main pathological basis of immune-type RSA patients is abnormal immune function. Helper T-cell 2 (Th2) cells secrete serum IL-4, which mainly mediates B-lymphocyte proliferation and antibody production and can protect pregnancy by inhibiting the activation of cellular responses such as NK cells and preventing secondary damage to the fetus from the response [25]. Th1 cells secrete serum IFN-*γ* to impede cell growth and embryonic development and result in pregnancy loss, and IFN-*γ* also activates macrophages and causes an inflammatory response [26]. In this study, by measuring the levels of factors such as IL-4 and IFN-*γ* in RSA patients before and after intervention, we found that the serum IL-4 level in the study group was higher than that in the control group after the intervention, and the IFN-*γ* level and IFN-*γ*/IL-4 ratio were lower than those in the control group, indicating that the integrated nurses-physicians collaboration intervention combined with low-molecular-weight heparin treatment could improve the immune function of the patients more effectively. Heparin is able to inhibit some cellular functions, improve coagulation disorders in patients, reduce damage to vascular endothelial cells, and thus regulate human immunity [27]. In addition, the patients' anxiety and depression improved significantly after the integrated medical and nursing interventions, and the level of sympathetic physiological arousal and endorphin level in the body could also improve the body's immune function to some extent; thus the study group improved even more [28]. The patients in the study group were all more satisfied with the intervention than the control group, indicating that the implementation of the integrated nurses-physicians collaboration model was significant in improving the relationship between physicians, nurses, and patients.

In conclusion, the application of nurses-physicians collaboration in the clinical treatment of immune-type RSA patients is effective. The application of this nursing model can significantly improve patients' psychological status, sleep quality, and immune function, reduce the incidence of adverse events, and is also important for the improvement of patients' pregnancy outcomes and the pulling together of the relationship between physicians, nurses, and patients.

## Figures and Tables

**Figure 1:** Comparison of pregnancy outcomes between the two groups. Compared with the control group for the success rate of fetal preservation, ^∧^*P* < 0.05.

**Figure 2:** Comparison of negative mood scores and sleep quality scores before and after intervention between the two groups. (a) Average SAS scores. (b) Average SDS scores. (c) Average PSQI scores. Compared with the same group before the intervention, ^*∗*^*P* < 0.05. Compared with the control group after intervention, ^∧^*P* < 0.05.

The article "Clinical Impact of Nurses-Physicians Collaboration Intervention on the Treatment of Immune Recurrent Spontaneous Abortion with Low-Molecular-Weight Heparin" was retracted in 2023. Reasons: unreliable results or conclusions; concerns about the data; concerns about the peer review; concerns about the citations.

**Figure 3:** Comparison of immune function indexes before and after intervention between the two groups. (a) Average IFN-*γ* levels. (b) Average IL-4 levels. (c) Average IFN-*γ*/IL-4 ratio. Compared with the same group before the intervention, ^*∗*^*P* < 0.05. Compared with the control group after intervention, ^∧^*P* < 0.05.

**Figure 4:** Comparison of patient satisfaction survey scores between the two groups. (a) Patient satisfaction with inpatient guidance. (b) Patient satisfaction with physicians. (c) Patient satisfaction with nurses. (d) Patient satisfaction with physician-nurse collaboration. (e) Patient satisfaction with doctor-patient communication. (f) Total satisfaction score. Compared with the control group, ^∧^*P* < 0.05.

**Figure 5:** Comparison of the incidence of adverse drug reactions between the two groups. Compared with the incidence of total adverse reactions in the control group, ^∧^*P* < 0.05.

**Table 1:** Comparison of general information between the study group and the control group.

Information	Control group (*n* = 47)	Study group (*n* = 47)	*P* value	
Age (*n*, %)	<25 years	7 (14.89)	8 (17.02)	0.975
	25∼30 years	18 (38.30)	19 (40.43)	
	31∼35 years	16 (34.04)	15 (31.91)	
	>35 years	6 (12.77)	5 (10.64)	
Miscarriage history (*n*, %)	2 times	24 (51.06)	26 (55.32)	0.916
	3 times	14 (29.79)	13 (27.66)	
	≥4 times	9 (19.15)	8 (17.02)	
Wedding time (*n*, %)	<5 years	10 (21.28)	12 (25.53)	0.755
	5∼10 years	23 (48.94)	24 (51.06)	
	>10 years	14 (29.78)	11 (23.40)	
Duration of pregnancy (*n*, %)	5∼7 weeks	21 (44.68)	20 (42.55)	0.974
	8∼10 weeks	17 (36.17)	18 (38.30)	
	11∼12 weeks	9 (19.15)	9 (19.15)	

## Data Availability

The data are available from the corresponding author upon request.
